RETRACTED

# The distribution and socioeconomic burden of Hepatitis C virus in South Australia: a cross-sectional study 2010–2016

**DOI:** 10.1186/s12889-019-6847-5

**Published:** 2019-05-08

**Authors:** Bernard Luke Edmunds, Emma Ruth Miller, George Tsourtos

**Affiliations:** Flinders University, GPO Box 2100, Adelaide, 5001 South Australia

**Keywords:** Hepatitis C, Epidemiology, Socio-economic status, Hepatitis C treatment

## Abstract

**Background:**

Hepatitis C virus infection (HCV) is a communicable disease of increasing global importance with 1.75 million new infections and 400,000 related deaths annually. Until recently, treatment options have had low uptake and most infected people remain untreated. New Direct Acting Antiviral medications can clear the virus in around 95% of cases, with few side-effects. These medications are restricted in most countries but freely accessible in Australia, yet most people still remain untreated. This study applies a cross-sectional research design to investigate the socio-spatial distribution of HCV in South Australia, to identify vulnerable populations, and examine epidemiological factors to potentially inform future targeted strategies for improved treatment uptake.

**Method:**

HCV surveillance data were sourced from South Australia’s Communicable Diseases Control Branch and socio-economic population data from the Australian Bureau of Statistics from January 2010 to December 2016 inclusive. HCV cases were spatially mapped at postcode level. Multivariate logistic regression identified independent predictors of demographic risks for HCV notification and notification source.

**Results:**

HCV notifications (*n* = 3356) were seven times more likely to be from people residing in the poorest areas with high rates of non-employment (75%; *n* = 1876) and injecting drug use (74%; *n* = 1862) reported. Notifications among Aboriginal and Torres Strait Islander people were around six times that of non-Indigenous people. HCV notifications negatively correlated (Spearman’s rho − 0.426; *p* < 0.001) with socio-economic status (residential postcode socio-economic resources Index). History of imprisonment independently predicted HCV diagnoses in lesser economically-resourced areas (RR1.5; *p* < 0.001). Independent predictors of diagnosis elsewhere than in general practices were non-employment (RR 4.6; *p* = 0.028), being male (RR 2.5; p < 0.001), and younger than mean age at diagnosis (RR 2.1; *p* = 0.006).

**Conclusions:**

Most people diagnosed with HCV were from marginalised sub-populations. Given general practitioners are pivotal to providing effective HCV treatment for many people in Australia a most concerning finding was that non-employed people were statistically less likely to be diagnosed by general practitioners. These findings highlight a need for further action aimed at improving healthcare access and treatment uptake to help reduce the burden of HCV for marginalised people, and progress the vision of eliminating HCV as a major public health threat.

RETRACTED

## Background

An estimated 80 million people live with active hepatitis C virus infection (HCV) worldwide [1], with approximately 1.75 million new infections and 400,000 related deaths annually [2]. In developed countries, HCV antibody prevalence ranges from 0.1 to 1.1% [3]. This is in part due to the relatively high chronicity of infection (approximately 75% of those infected [4–8]) and low access to effective treatment [9–12]. Non-treatment typically results in the development of hepatic fibrosis which may lead to cirrhosis and hepatocellular carcinoma; with related mortality occurring decades after infection [4, 5, 8, 12]. Until recently, HCV treatments globally have been expensive, poorly tolerated, and of low curative potential such that most chronically infected people remain untreated [9–12].

HCV treatments were recently transformed with Direct Acting Antiviral medications (DAAs) providing superior regimens, lower toxicity, and virus clearance in around 95% of cases [9, 11, 13–17]. Yet most countries do not offer affordable access to DAAs due to prohibitive expense [9, 18–20] and only around 7 % of people diagnosed with HCV globally have received treatment [2]. In response to issues with low treatment uptake, the World Health Organization (WHO) is urging action to ensure DAAs are affordable and accessible to people who need them; with the aim of eliminating viral hepatitis as a public health threat by the year 2030 [9, 21].

In developed countries, HCV is largely transmitted through injecting drug use (IDU) [9, 22–31]. High infection rates, poorer prognosis and burden of disease have been associated with lower socio-economic status (SES) [32–38]. Greater frequency of IDU and higher HCV prevalence is associated with lower income [33, 36, 37, 39], lower education attainment [25, 33–37, 39–42], reduced employment [33, 34, 42–44] and homelessness [45–53]. Conversely, higher education level and higher paid occupation are both associated with increased knowledge of HCV [54] and decreased HCV prevalence [25]. Furthermore, people living with HCV commonly perceive and report discrimination [55–60], with those from disadvantaged and marginalised backgrounds less likely to access treatments compared to the overall population [38, 61, 62]. This can result in regional differences in HCV prevalence along the social gradient as has been observed in some areas of Holland [63], France [64], Scotland [65], United States of America [39], and China [66]. Yet, apart from these studies, there have been few attempts to define the burden of HCV morbidity in relation to SES in most areas, including South Australia (SA) [67].

RETRACTED

In Australia, HCV prevalence is estimated at around 1 % [3], with approximately 230,000 HCV cases, of whom 75% are diagnosed [12, 68]. Although DAAs remain largely inaccessible in most countries, affordable access has been available in Australia since March 2016 through Government subsidy [9, 18, 19, 69]. Furthermore, in 2016 prescribing regulations were reformed in Australia enabling the majority of patients with less complicated chronic HCV infections to be treated by general practitioners in the community. This was followed by further reform allowing nurse practitioners to prescribe DAAs in 2017 [70–72].

Following these advancements, HCV treatment uptake in Australia has improved from a low of 2% for interferon-based therapies; yet has only increased to 20% with roll-out of the latest DAAs [12]. Thus, despite providing what is considered to be a leading model for chronic HCV treatment [73], the majority of people infected with HCV in Australia remain untreated [12, 73]. With the current treatment uptake, HCV related liver disease in Australia is projected to triple by 2030 [11].

Research revealing patterns in HCV epidemiology may potentially better inform targeted public health interventions to reach greater numbers of people living with chronic HCV infection, improve DAA treatment uptake, and eradicate unnecessary HCV burden [21, 74]. This study aimed to investigate the socio-spatial distribution of newly diagnosed HCV in South Australia and identify vulnerable populations. Potentially, this information will guide the development of appropriately targeted strategies with which to improve treatment uptake among a population of people who have affordable access to DAAs. As such, our research may be considered an international bellwether for the scale-up of DAAs and for the control of HCV epidemics in developed countries.

## Methods

### Study design, population and setting

We conducted a cross-sectional analysis of all people newly notified with HCV in SA from January 2010 to December 2016 inclusive. SA has a population of approximately 1.7 million, with a median age of 39.8 years. Of these, 22% of people report being born overseas and 2% identify as being an Indigenous Australian [75]. A great proportion of SA’s population, around 1.3 million people, are clustered in and around the capital city Adelaide [75].

Mandated surveillance of HCV commenced in most Australian jurisdictions in 1997, including SA [76] where the data for the current analysis has been sourced. SA’s Department of Health and Ageing Communicable Disease Control Branch (CDCB) obtains HCV notifications under State legislation [77, 78] via an advanced population surveillance dual notification system in which laboratory and diagnosing medical practitioners provide information on each episode of infection, using nationally agreed case definitions for classifying HCV [79].

RETRACTED

De-identified HCV surveillance data were sourced from the CDCB and Socio-economic Index for Areas (SEIFA) data was sourced from the Australian Bureau of Statistics (ABS) 2011 Australian Census. SEIFA is a measure used by the ABS to rank communities in Australia based on their socio-economic status (SES). Higher decile scores are associated with higher SES. In total, there were 3656 HCV cases notified to the CDCB over the study period. SEIFA data included 1,591,731 respondents from SA [80] with a participation rate of 98.3% of the total State population. CDCB and SEIFA data were acquired by mandate of the Commonwealth of Australia and the SA Government under State and Federal legislation [77, 78, 81].

### The datasets

We abstracted HCV surveillance data for all SA notifications between January 2010 and December 2016 inclusive. Cases were identified by testing positive to HCV antibody (anti-HCV) or ribonucleic acid (RNA) amplification test (HCV-RNA polymerase chain reaction [PCR]) for the first time [82]. All cases were defined according to the Communicable Disease Network of Australia hepatitis C case definitions [83]. Notified cases were certified as ‘Newly acquired’ infections if an individual had tested positive for HCV within 24 months of a negative test; or presented with clinical signs of acute hepatitis in conjunction with a positive anti-HCV or RNA test [82, 83]. All other notifications were categorised as ‘Unspecified’. Ethics approval was granted by the SA Department for Health and Ageing Human Research Ethics Committee (Government of South Australia).

SEIFA data were derived from the compulsory census completed by all residents of SA on the 9th August, 2011. The SEIFA includes four indices that indicate differing collective socio-economic characteristics of people living within postal areas. All four SEIFA indices formed part of this analysis. The Indices differ in that the Index of Relative Socio-Economic Disadvantage indicates the proportion of relatively disadvantaged people in that area; the Index of Relative Socio-Economic Advantage and Disadvantage indicates ranks on a continuum of most disadvantaged to most advantaged; the Index of Economic Resources (IER) summarises variables relating to financial aspects of relative socio-economic advantage and disadvantage; and the Index of Education and Occupation summarises variables relating to the educational and occupational aspects of relative socio-economic advantage and disadvantage [84]. The ABS broadly define socio-economic advantage and disadvantage in relation to access to material resources, social resources and participation in society [84].

RETRACTED

The census survey was self-completed by households and represented all persons present in the residence on that night. ABS Census Collectors were responsible for survey delivery and collection at all dwellings; and supporting homeless people to complete the survey. Collectors were allocated computer-generated areas without overlap or omission. Clear instructions for survey completion were provided by Collectors, complemented by a national media information campaign, and efforts made to assist people from non-English speaking backgrounds. The survey could be completed online or in print [85].

### Analysis

The statistical analysis involved three stages. Descriptive analyses were used to check for possible errors in the data, establish if certain variables were normally distributed, calculate measures of central tendency, and help identify risk factors. The second stage involved bivariate analyses, the results of which informed what variables would be entered as independent variables in the third stage: multivariate logistic regression modelling.

Spatial analyses were undertaken by merging HCV surveillance postcode data with SEIFA using ABS 2011 Census Postal Area boundaries to enable spatial mapping at the postal area level (using ArcGIS version 10.4.1). In total, there were 3411 notifications for which SA residential postcode and SEIFA rankings could be merged. SEIFA Index deciles were then established for every postcode, enabling the ranking of postcodes according to SEIFA Index. We undertook correlation analyses via Spearman’s Rho and Chi square tests to determine significant relationships between HCV notifications and major demographic risks, calculating rate ratios and rates of difference.

Collinearity was assessed using Chi-Square and Phi statistics in relation to building five multivariate binomial models. Category by category interaction for sex and IDU in logistic regressions was initially tested and goodness of fit was tested using the Hosmer-Lemeshow test. In sensitivity analyses we also tested interactions between each exposure variable of interest and sex, as well as for IDU behaviour in the past 2 years for all models excluding model 3, which had IDU risk behaviour as the outcome. Injecting drug use was more likely in males in older age groups, however no other significant interactions were found.

RETRACTED

The first model aimed to establish the association between area of residence and HCV notifications using SIEFA Indices dichotomised at the median. SEIFA IER was used as the dependent variable to explore the social distribution of HCV notifications (because the correlation between IER HCV notifications was the strongest relative to other indices). Explanatory variables were statistically significant demographic and risk factors identified through bivariate analysis.

The second and third models aimed to identify independent predictors among statistically significant risk factors identified through bivariate analysis (non-employment and IDU history respectively were the dependent variables). Explanatory variables were statistically significant demographic and risk factors that were identified through bivariate analysis; except where these were the same as the dependent variable (non-employment for Model 2 and IDU history for Model 3). With 98% (n. 300) of people with a history of imprisonment being non-employed, the history of imprisonment explanatory variable was excluded from the second model.

Models four and five aimed to identify independent predictors of accessing general practitioner for vulnerable sub-populations. A binary of general practitioner and State Government notification source was the dependent variable with vulnerable sub populations the explanatory variables (IDU < 2 years, employment, indigenous status, Australian origin and age of first IDU dichotomized at the median). The fourth model included all notifications while the fifth model excluded notifications from prison health services, as these people are incarcerated and unable to access public hospitals and general practitioners. All models included potential confounding variables (such as age dichotomised at the median, sex and Australian origin). Missing data were excluded from all statistical analyses, which were undertaken using Stata (release 15, Stata Corporation, College Station, TX, USA).

## Results

### Descriptive analysis

During the period 2010 to 2016 there were 3656 notifications, of which 91% (*n* = 3329) were cases of unspecified duration and 9% of infections (*n* = 327) were classified as newly acquired. Annual frequencies of HCV notifications remained relatively stable over the seven-year period ranging from 495 in 2014 to 538 in 2013 and 2016 (Fig. 1). Age was normally distributed for both males and females with a greater proportion of notifications among males (63%). Data relating to Indigenous status were missing for 2520 notifications (69%), with 147 (13%) HCV notifications identified as Indigenous Australian. Seven hundred people (22%) were reported to have been born outside Australia (460 missing; 13%). Australia was the main reported country of birth (78%, *n* = 2496), followed by the United Kingdom and Ireland (2.7%, *n* = 86), and Vietnam (2.6%, *n* = 83). For the frequencies of reported potential HCV risk factors see Table 1.

RETRACTED

**Fig. 1:** HCV Notifications for South Australia 2010–2016

**Table 1:** Descriptive statistics for HCV Notifications in South Australia 2010–2016

*Identified Risk Factors* ^*a*^	*Unspecified Notifications (%)*	*Notifications < 24 months (%)*	*Total (%)*
Non-Employment	1642 (75%)	225 (90%)	1867 (77%)
Injecting Drug Use	1578 (72%)	284 (90%)	1862 (74%)
Injecting drug use in previous 24 months	1257 (57%)	275 (87%)	1532 (61%)
Birth outside Australia	683 (23%)	17 (5%)	700 (22%)
Prison history	432 (33%)	91 (45%)	523 (35%)
Tattoos	414 (35%)	69 (35%)	483 (35%)
Household Contact	149 (13%)	51 (26%)	200 (15%)
Indigenous Australian	120 (12%)	27 (28%)	147 (13%)
Healthcare related exposure	137 (11%)	1 (0.5%)	138 (10%)
Opposite-sex partner infected with HCV	94 (8%)	34 (17%)	128 (9%)
Blood Products (Outside Australia)	57 (5%)	- (0%)	57 (4%)
Blood Products (Australia)	51 (4%)	1 (0.5%)	52 (4%)
Piercing (only from 2005)	49 (4%)	19 (10%)	68 (5%)
Needle Stick Injury (non HCW)	25 (2%)	13 (7%)	38 (3%)
Perinatal transmission	11 (1%)	1 (0.5%)	12 (0.9%)
Needle Stick Injury (HCW)	7 (0.6%)	2 (1%)	9 (0.7%)
Same-sex partner infected with HCV	3 (0.26%)	5 (3%)	8 (0.6%)
Notification Sources	*Male (%)*	*Female (%)*	*Total (%)*
Metropolitan General Practitioner	813 (35)	567 (42)	1380 (38)
Rural or Remote General Practitioner	387 (17)	256 (19)	643 (18)
Prison Health Services	295 (13)	47 (3)	342 (9)
Royal Adelaide Hospital	176 (8)	77 (6)	253 (7)
Flinders Medical Centre	91 (4)	67 (5)	158 (4)
Drug Alcohol Services Council	95 (4)	35 (3)	130 (4)
Lyell McEwin Hospital	70 (3)	51 (4)	121 (3)
Queen Elizabeth Hospital	67 (3)	39 (3)	106 (3)
Other Public Hospitals or Health Centres	79 (3)	37 (2)	116 (3)
Other not specified	56 (2)	46 (3)	102(3)
Government Aboriginal Health Service	34 (1)	26 (2)	60 (2)
Sexually Transmitted Diseases Clinic	43 (2)	16 (1)	59 (2)
Woman’s and Children’s Hospital	4 (0)	32 (2)	36 (1)
Modbury Hospital	14 (1)	11 (1)	25 (1)
Mental Health Services	18 (1)	12 (1)	30 (1)
Australian Red Cross Blood Service	16 (1)	14 (1)	30 (1)
Aboriginal Controlled Health Services	18 (1)	9 (1)	27 (1)
Private Hospitals	14 (1)	5 (0)	19 (1)
Repatriation General Hospital	7 (0)	5 (0)	12 (0)
Cross Border Notifications	7 (0)	0 (0)	7 (0)
TOTAL	2304 (100)	2352 (99)	3656 (99)

*HCV* Hepatitis C virus, *HCW* Health Care Worker

^a^Multiple risk factors reported

Notifications were most frequently received from general practitioners (primary care physicians) who notified HCV in 55% of cases (*n* = 2023), with 38% (*n* = 1380) from metropolitan areas (see Table 1). Notifications from major metropolitan hospitals were 18% for males (*n* = 404) and 19% for females (*n* = 266). Notifications from Prison Health Services were greater for males 13% (*n* = 295) than females 3% (*n* = 47). Prison Health Services notifications were highest among Indigenous Australians, constituting 27% of notifications. Thirty-seven percent of Indigenous Australian male notifications (n = 29) and 16% of Indigenous Australian female notifications (*n* = 11) were received from the Prison Health Service.

RETRACTED

### Descriptive statistics: spatial distribution

Of 319 SA postal areas for which SEIFA rankings and HCV notifications could be merged, 245 residential postcodes had HCV notifications (77%) with a median number of three (IQR 12). Thirty-seven percent (*n* = 1273) of notifications resided in the lowest 10% of IER postcodes (median 21; IQR 40) and 60 % (*n* = 2040) resided in the lowest 20% of IER postcodes. Conversely, 1 % (*n* = 42) of notifications resided in the highest 10% of IER postcodes (median 1; IQR 3). HCV notifications therefore were seven times more likely to be from people residing in the least economically-resourced 10% of postcodes, and 20 times more likely compared to people living in the wealthiest deciles.

Rural residential postcodes with greater than 50 notifications were in the areas of Murray Bridge (2.9%; *n* = 107), Mount Gambier (2.9%; n = 107), Port Augusta (2.2%; *n* = 81) and Port Lincoln (1.7%*n* = 62). These communities represent locations of four SA Prisons outside the Adelaide metropolitan area. Prison Health Services notification source, which accounted for 9% (*n* = 342) of total notifications, were of greater frequency in these areas. Notifications in Adelaide’s metropolitan postcodes were greatest in the Adelaide Central Business District (CBD; 4.2%; *n* = 155) and Enfield/Northfield (3.4%; *n* = 123); both areas have the largest prison populations. Prison Services notifications in these postcodes were 38% (*n* = 49) and 64% (*n* = 74) respectively.

Greater numbers of notifications were also clustered in the northern suburbs of the Adelaide metropolitan area, an area that has lower socio-economic levels than elsewhere in SA. Specifically, these were Salisbury (3.1% *n* = 114), Elizabeth (3% *n* = 112), Davoren Park (2.6% *n* = 96) and Blakeview/Andrews Farm (1.7%*n* = 63). With Prison Health Services notifications excluded from spatial analysis to reflect the broader community (see Fig. 2), the proportion of notifications clustered in these northern suburbs increased relative to other postcodes. A greater proportion of notifications were also recorded in the Adelaide CBD (*n* = 155; 4%). In this area HCV notifications had a lower mean age of 39 years (SD = 10; t-test *p*-value =0.002), a greater male population (*n* = 134;86%; t-test p-value < 0.001) and the highest rates of non-employment (*n* = 53; 87%; t-test p-value < 0.001), IDU (*n* = 58; 85%; t-test p-value < 0.001) and history of imprisonment (*n* = 10; 40%; t-test p-value < 0.001) for any postcode in SA.

RETRACTED

**Fig. 2:** Number of non-Prison Health Service HCV Notifications per Postal Area in South Australia’s Metropolitan area (map generated using ArcGIS version 10.4.1)

### Bivariate analysis

All four SEIFA Indices were found to correlate negatively with HCV postcode notification numbers with the correlation stronger for the IER (Spearman’s Rho − 0.422; *p* < 0.001). The correlation between HCV notifications and the IER was strongest among Indigenous Australian males (Spearman’s Rho − 0.611; p < 0.001) followed by Indigenous Australian females (Spearman’s Rho − 0.598; p < 0.001), total females (Spearman’s Rho − 0.422; p < 0.001) and then males (Spearman’s Rho − 0.414; p < 0.001).

Non-employment, IDU and Prison Services contact were significantly associated with people of Australian origin, regardless of Indigenous status (Table 2). Birth outside of Australia was significantly associated with healthcare related infections and household contact. History of imprisonment, non-employment, IDU and being an Indigenous Australian were significantly associated with residence in lower economically-resourced postcodes (<= median IER score of 2; *p* < 0.001). Additionally, needle-stick injury among healthcare workers, having received blood products in Australia, healthcare related exposure and tattoos were significantly associated with residence in greater economically-resourced postcodes (> median IER score of 2; *p* < 0.05: see Table 3).

**Table 2:** Bivariate analysis of HCV Notifications and Demographic Risks in South Australia 2010–2016

	Rate ratio (95%CI)	Rate difference (95%CI)	*p*-Value*
Non-Employment			
Indigenous Australian	5.04 (1.25–20.33)	0.14 (0.07–0.21)	0.007
Female	1.14 (1.00–1.29)	0.05 (0.00–0.09)	0.048
Australian origin^a^	1.11 (1.04–1.17)	0.08 (0.03–0.12)	< 0.001
IDU previous 24 months			
Indigenous Australian	3.53 (2.32–5.35)	0.13 (0.10–0.17)	< 0.001
Australian origin	1.58 (1.49–1.67)	0.34 (0.31–0.37)	< 0.001
Male	1.45 (1.36–1.55)	0.26 (0.22–0.31)	< 0.001
Injecting Drug Use			
Indigenous Australian	4.93 (2.54–9.57)	0.13 (0.09–0.16)	< 0.001
Australian origin	2.03 (1.87–2.22)	0.47 (0.42–0.51)	< 0.001
Male	1.14 (1.06–1.22)	0.08 (0.04–0.12)	< 0.001
Prison Services contact			
Indigenous Australian	3.93 (2.57–6.04)	0.21 (0.14–0.28)	< 0.001
Australian origin	1.52 (1.44–1.61)	0.33 (0.29–0.36)	< 0.001
Male	1.45 (1.36–1.55)	0.26 (0.22–0.31)	< 0.001
Tattoo			
Male	1.21 (1.12–1.31)	0.13 (0.08–0.18)	< 0.001
Australian origin	1.43 (1.34–1.53)	0.27 (0.22–0.31)	< 0.001
Household contact			
Female	1.66 (1.42–1.94)	0.21 (0.14–0.29)	< 0.001
Origin outside Australia	1.22 (1.13–1.31)	0.15 (0.09–0.21)	< 0.001
Healthcare related infection			
Origin outside Australia	2.23 (1.86–2.66)	0.31 (0.22–0.40)	< 0.001
Female	1.48 (1.23–1.78)	0.16 (0.07–0.25)	< 0.001
Blood products (outside Australia)			
Female	1.37 (1.04–1.83)	0.13 (− 0.00–0.26)	0.045

*IDU* Injecting Drug Use, *HCW* Health Care Worker, *HCV* Hepatitis C virus

^*^Tested using chi square

^a^Australian origin includes Aboriginal and Torres Strait Islander people

RETRACTED

**Table 3:** Bivariate analysis of HCV Risks and SEIFA Economic Resources Index in South Australia 2010–2016

	Rate ratio (95%CI)	Rate difference (95%CI)	*p*-Value*
HCV and SEIFA IER Post Codes <= median score (2)			
History of imprisonment	1.55 (1.44–1.66)	0.29 (0.25–0.34)	**< 0.001**
Non-Employment	1.33 (1.21–1.46)	0.16 (0.11–0.20)	**< 0.001**
IDU previous 24 months	1.30 (1.21–1.39)	0.15 (0.11–0.19)	**< 0.001**
Injecting Drug Use	1.20 (1.10–1.30)	0.11 (0.06–0.15)	**< 0.001**
Indigenous Australian	1.24 (1.11–1.39)	0.15(0.07–0.23)	**< 0.001**
Sex partner same sex HCV	1.22 (0.82–1.84)	0.14 (− 0.16–0.44)	0.419
Perinatal	1.09 (0.73–1.63)	0.06 (− 0.21–0.32)	0.692
HCV and SEIFA IER Post Codes >median score (2)			
Needle Stick Injury (HCW)	2.27 (1.73–2.97)	0.49 (−0.26–0.72)	**0.005**
Blood Products in Australia	1.57 (1.24–1.98)	0.22 (0.08–0.35)	**0.001**
Healthcare related exposure	1.36 (1.14–1.63)	0.136 (0.05–0.22)	**0.002**
Tattoos	1.26 (1.10–1.44)	0.09 (− 0.38–0.15)	**< 0.001**
Needle Stick Injury (non-HCW)	1.29 (0.94–1.80)	0.114 (− 0.05–0.28)	0.154
Piercing (only from 2005)	1.22 (0.94–1.59)	0.09 (−0.38–0.21)	0.167
Blood Products (not Australian)	1.20 (0.90–1.61)	0.08 (−0.05–0.21)	0.237
Sex partner (opposite sex) has HCV	1.17 (0.95–1.44)	0.065(−0.03–0.16)	0.154
Australian origin^a^	1.09 (0.99–1.21)	0.04 (−0.01–0.08)	0.088
Household Contact	1.05 (0.87–1.26)	0.19 (−0.06–0.09)	0.615

Bold type indicates statistical significance at *p*-value < 0.05

*IDU* Injecting Drug Use, *HCW* Health Care Worker, *HCV* Hepatitis C virus

^*^Tested using chi square

^a^Australian origin includes Aboriginal and Torres Strait Islander people

### Multivariate analysis

The first multivariate model (Table 4) found a history of imprisonment, employment and female sex to independently predict residence in the lowest two SEIFA IER postcodes. The finding of greater employment in the lowest two SEIFA IER postcodes (RR 1.54) is explained by the high non-employment rate of 98% among people with a history of imprisonment disproportionately represented in the lowest two SEIFA IER postcodes (RR 1.54).

RETRACTED

**Table 4:** Multivariate Analysis of HCV Notifications in South Australia 2010–2016

	Rate ratio (95%CI)	Rate difference (95%CI)	*p*-Value^*^
MODEL 1: HCV notifications in low SEIFA IER postal areas (<= median; *n* = 3409)^#^			
History of imprisonment	1.54 (1.11–2.14)	0.23 (0.00–0.45)	**0.010**
Employment	1.54 (1.27–1.87)	0.18 (− 0.01–0.38)	**< 0.001**
Female	1.02 (1.01–1.02)	−0.01(− 0.18–0.16)	**< 0.001**
Non-Indigenous	1.16 (0.86–1.57)	0.15 (− 0.07–0.36)	0.322
Injecting Drugs last 2 years	1.16 (0.82–1.63)	−0.12 (− 0.08–0.33)	0.397
Younger than median age (42)	1.13 (0.84–1.53)	−0.05 (− 0.13–0.24)	0.421
MODEL 2: Non-employment notifications (*n* = 2425)^#^			
Injecting drugs last 2 years	1.37 (0.18–1.59)	0.18 (0.05–0.31)	**< 0.001**
Non-Australian origin	1.27 (1.17–0.14)	0.08 (− 0.05–0.29)	**< 0.001**
Younger than mean age (42)	1.28 (1.07–1.41)	0.14 (− 0.03–0.24)	**0.003**
Indigenous Australian	1.18 (1.09–0.28)	0.13 (0.06–0.20)	**< 0.001**
Female Sex	1.04 (1.04–1.04)	0.02 (− 0.02–0.02)	**< 0.001**
MODEL 3: IDU notifications (*n* = 3311)^#^			
Australian origin	3.51 (1.70–7.24)	0.51 (0.37–0.66)	**0.001**
History of imprisonment	1.56 (1.28–1.91)	0.31 (0.18–0.44)	**< 0.001**
Older than mean age (42)	1.12 (1.04–1.20)	0.02 (− 0.02–0.03)	**0.002**
Indigenous Australian	1.14 (1.06–1.23)	0.11 (0.05–0.17)	**< 0.001**
Male Sex^a^	1.06 (1.06–1.06)	0.02 (0.02–0.02)	**< 0.001**
Non-employment	1.18 (0.82–1.70)	0.15 (0.03–0.27)	0.367

Bold type indicates statistical significance at *p*-value < 0.05

*IDU* Injecting drug use

^*^Tested via binomial logistic regression

^#^Hosmer-Lemeshow test *p*-value > 0.05

^a^only in males aged older than 42 years.

The second and third multivariate models (Model 2 and Model 3; Table 4) identified independent predictors of statistically significant risk factors. The second model found independent predictors of non-employment among people newly diagnosed with HCV were (in rank order): injecting drugs in the previous 2 years, birth outside of Australia, being younger than 42 years of age, being an Indigenous Australian and being female. The third model found factors independently associated with IDU among people newly diagnosed with HCV were: Australian origin, a history of imprisonment, age older than 42 years and being an Indigenous Australian. Being male also independently predicted IDU exposure but sensitivity analyses indicated that this was only in those aged older than 42 years. Notifications from those reporting birth in Australia were more than three and a half times more likely to report IDU history compared to those originating from outside Australia.

RETRACTED

The fourth model (Model 4; Table 5) identified predictors of notification source to investigate patterns of access to general practitioners. Prison Health Services notifications were then removed to test notifications in the broader community who were more able to access general practitioners. With these removed in the final model non-employed people, males, and people younger than 42 years of age were over 30% less likely to attend general practitioners for HCV diagnosis (Model 5; Table 5).

**Table 5:** Multivariate Analysis of HCV Notification Source in South Australia 2010–2016

	Rate ratio (95%CI)	Rate difference (95%CI)	*p*-Value*
MODEL 4 State Government (non-General Practitioner) notification source *(n = 3460)* ^#^			
Non-employment	4.88 (1.27–18.86)	0.37 (− 0.21–0.53)	**0.021**
Male Sex	2.31 (1.50–3.57)	0.41 (0.26–0.55)	**< 0.001**
Age at diagnosis < median (42)	1.99 (1.25–3.17)	0.36 (0.20–0.51)	**0.004**
Indigenous Australian	1.20 (1.04–1.38)	0.09 (− 0.01–0.19)	**0.012**
IDU < 2 years	1.17 (1.02–1.35)	0.08 (0.08–0.08)	**0.028**
Age first IDU < median (20)	1.10 (1.10–1.10)	0.07 (0.07–0.07)	**< 0.001**
Australian origin	1.06 (0.93–1.23)	− 0.05 (− 0.05–0.05)	0.38
MODEL 5 State Government (non-General Practitioner) notification source; Non-Prison Health Service (*n* = 3118)^#^			
Non-employment	4.61 (1.18–17.94)	0.34 (0.17–0.51)	**0.028**
Male Sex	2.46 (1.49–4.06)	0.34 (− 0.18–0.51)	**< 0.001**
Age diagnosed < mean (42)	2.05 (1.23–3.41)	0.31 (0.14–0.47)	**0.006**
Age first IDU < median (20)	1.13 (1.13–1.13)	0.05 (0.05–0.05)	**< 0.001**
Australian origin	1.08 (0.66–1.78)	− 0.06 (− 0.06—0.06)	0.75
Indigenous Australian	1.23 (0.98–1.71)	0.10 (− 0.17–0.36)	0.069
IDU < 2 years	1.29 (0.98–1.71)	0.09 (0.09–0.09)	0.07

Bold type indicates statistical significance at *p*-value < 0.05

*IDU* Injecting drug use

^*^Tested via binomial logistic regression

^#^Hosmer-Lemeshow test with *p*-value > 0.05

## Discussion

This is the first study to examine spatial distribution and socio-economic burden of HCV at a population level in Australia, and one of a few published studies investigating this topic worldwide. Despite the recent introduction of affordable access to DAAs in Australia, most people with chronic HCV infection remain untreated. Such research is necessary to locate and understand areas with higher burden of disease, more effectively target interventions and improve treatment uptake.

RETRACTED

### Inequitable distribution

In our study disproportionately high frequencies of HCV notifications were found to cluster in particular areas; a phenomenon consistent with research undertaken in Holland [63], United States of America [39], and China [66]. Our results indicate HCV is inequitably distributed across SA with most notifications arising in the least economically resourced areas. HCV notifications were seven times more likely in people residing in the poorest areas compared to the State mean and 20 times more likely compared to the greatest economically resourced postcodes.

This inequitable distribution of HCV notifications may be explained, at least in part, by multiple layers of disadvantage occurring lower down the social gradient [86]. Sub-populations found to be vulnerable to HCV infection in this study included PWID, non-employed people, people with history of imprisonment, and Indigenous Australians. Our research identified these vulnerable populations disproportionately reside in the least economically resourced postcodes in South Australia. The socio-spatial distribution of HCV cases in SA that we revealed clearly identifies areas of greatest need for enhanced DAAs treatment uptake strategies.

The inner-city area of Adelaide was anomalous with a high frequency of HCV notifications despite increased SEIFA Index scores in comparison to other cluster areas. This may be related to the younger age, larger male population and higher proportions of non-employment, IDU, and history of imprisonment observed in this area. These are risks associated with homelessness [46, 47, 87–89] which is linked to higher rates of HCV infection in Australia, Canada, the United Kingdom and United States of America [45–53]. As the greatest concentration of homeless people in SA reside in this postcode [90] further investigation into homelessness and HCV in this area may potentially inform targeted treatment strategies.

### Injecting drug use

The proportions of cases reporting IDU as an HCV risk factor (90% of newly acquired cases and 72% of cases of unspecified duration) was comparable to those reported elsewhere in Australia during the same period, and higher than early findings in Australia of around 60–70% during the 1990’s [74, 91, 92]. The high proportion of PWID observed among newly diagnosed cases of HCV has implications for healthcare access and treatment uptake. People living with HCV often face stigma and discrimination associated with IDU [55–60, 65]. This occurs in health care settings and can result in reduced intention by people to engage with HCV treatments [55–60] or exclusion from HCV treatment by practitioners on the basis of IDU [71, 93, 94].

RETRACTED

IDU among HCV notified cases in this study were also independently predicted by non-employment, a history of imprisonment, and being an Indigenous Australian. These findings illustrate the concept of multiple stigma, where people experience stigma on various concurrent levels [57, 95, 96]. This has been linked to health inequities [96] and may assist in explaining why disadvantaged and marginalised people living with HCV are significantly less likely to access treatments [38, 61, 62]. Our findings support dedicated HCV screening and treatment strategies intended for PWID in SA, with focused testing shown to be cost-effective in all settings [97–100].

### Non-employment

Most notified cases of HCV were not in paid employment with higher proportions of non-employment in Adelaide’s CBD and the northern Adelaide metropolitan area where HCV notification frequencies were the greatest and economic-resources most limited. This has likely implications for HCV treatment uptake with unemployment both a determinant of poorer health and a barrier to treatment [86, 101–107].

Few studies have explored healthcare access and HCV treatment uptake among non-employed or socioeconomically disadvantaged people and findings are mixed. A French study in an area with good primary care affordability found geographical proximity to general practitioner, rather than socioeconomic context of neighbourhood, was the main factor limiting hepatitis C detection [64]. Conversely, in Scotland strong associations were found between HCV detection and socioeconomic deprivation, with less convincing evidence for a measure of travel-time to the nearest general practitioner [65]. As we found a large proportion of non-employed people newly notified with HCV were less likely to access general practitioners in Australia, further research to understand this is warranted.

### Prison history

The high proportion of HCV cases reporting past imprisonment in our study is consistent with trends identified in the literature reporting high HCV prevalence in prison settings [30, 74, 108–111], and particularly high among Indigenous Australians and female prisoners [109, 111–118]. Almost all notifications with history of imprisonment in this study reported non-employment, past IDU, and residence in lesser economically resourced postal areas; with Indigenous Australians significantly overrepresented. Theoretically, prison settings are therefore well placed to facilitate treatment access and uptake for a large number of identified vulnerable populations.

Prison settings are also well-placed for meeting the WHO objectives for focused testing and treatment services [119]. In prison settings the HCV treatment cascade can be supported by a single treating team using the continuous process of awareness, testing, referral, disease stage assessment, treatment initiation and monitoring [9]. One example of how this process might be established is described in the SA Government’s Prisoner Blood Borne Virus Prevention Action Plan 2017–2020 [120]. This action plan has potential to decrease the burden of HCV identified in vulnerable populations with disproportionate history of imprisonment in SA.

RETRACTED

### Indigenous status

With Indigenous Australians constituting around 2% of the SA population [75], HCV notifications for Indigenous Australians were over six times that of non-Indigenous people. This is higher than previously reported in Australia [82, 106, 107], and may reflect geographical differences in risk behaviours [20]. This inequity may be explained by structural or social factors influencing position on the social gradient of health [38, 86, 121]. This has been associated with constitutional and democratic exclusion [122–125], disempowerment through protection and assimilation policies [32, 126–128], and economic marginalisation [129–131]; which has reinforced racism and resulted in public health inequities [122, 132–135]. It is widely accepted for this to improve a focus on addressing social determinants of health (SDH) is necessary [135–140]. This aligns with similar findings among First Nations people in Canada where understanding the underlying contextual socioeconomic factors driving this inequity is considered essential [141, 142].

To address health inequities that are influenced by structural or social factors it is important for health promotion strategies to extend beyond traditional behaviour-change approaches [104, 122, 143–147]. It is widely accepted that addressing the underpinning SDH is crucial to correcting health inequities experienced by Indigenous Australians [116, 135–138, 140]. As Indigenous populations are known to have been excluded from healthcare services due to discrimination, or services that are not sensitive to cultural differences, specific culturally appropriate approaches are clearly needed to improve HCV screening and DAAs treatment uptake among Indigenous Australians [2, 116, 148–153].

### Access to healthcare

That non-employed people, males and younger people with HCV are significantly less likely to be notified by general practitioners has important implications for HCV treatment. Most people in Australia receive primary health care through general practitioners, and current HCV models of care are largely reliant on general practitioners for disease stage assessment, treatment initiation and monitoring (or in more complex cases, referral to specialist physicians) [70, 71]. Improving access to general practitioners and supporting general practitioners to initiate treatment are therefore important factors for improving DAAs treatment uptake [70, 71].

RETRACTED

Additional approaches may also be necessary to effectively target, engage, screen and provide treatment for the vulnerable populations we’ve identified who may be experiencing barriers to accessing general practitioners. Among these may include Indigenous Australians, PWID and people from lesser economically-resourced areas. Marginalised people commonly perceive and report discrimination [55–60] which can result in reduced intention to disclose HCV status or risks and hinder engagement in treatment [55–60]. People experiencing difficulties accessing treatment via general practitioners may benefit from nurse-practitioner models of care which have recently been enhanced with authority to prescribe DAAs in some countries [154, 155], including in Australia from June 2017 [72].

Further research is recommended to design, implement and evaluate future interventions aimed at improving DAAs treatment uptake among the vulnerable populations we have identified. Specifically, a qualitative methodological approach is necessary to understand barriers to accessing DAAs treatment, barriers to treatment initiation by general practitioners, and alternative approaches that may be more practical or culturally appropriate for identified vulnerable populations. Models that have successfully improved HCV screening and treatment uptake for marginalised people elsewhere have involved threshold targeted Primary Health Care Services, Mobile Medical Clinics, HCV screening in hospital Emergency Departments, rapid diagnostic testing and point of care testing [56, 156–160].

### Limitations

Data for the current analysis were derived from a passive surveillance system, and therefore only known cases are included. With an estimated 25% of HCV cases undiagnosed in Australia (*n* = 57,617) [12], it is certain that cases were missed in this study. Given these cases have not accessed healthcare services for HCV testing it is plausible that the results of this study relating to disadvantaged and marginalised sub-populations are underestimated. One ameliorating factor is that we analysed a large state-wide database from which, consistent with our aims, we were able to identify those sub-populations contributing most to the notified cases in SA.

Notified cases classed as ‘newly acquired’ are established infections of less than 24 months duration. For this classification, it is necessary for cases to present for HCV screening; and then represent for re-screening within the 24-month period. That people re-present for testing so quickly suggests either a self-perception of greater risk of infection or an opportunity presents for re-testing. Such examples may include re-presenting on the occasions of sharing injecting equipment or on re-entry to prison; with both IDU and history of imprisonment risks particularly high in comparison to unspecified notifications. Subsequently some risk factors for ‘newly acquired’ data may be over-reported.

RETRACTED

Although ABS Postal Areas are the closest possible approximation of State Postcodes, there may be minor differences in ABS Postal Area and State Postcode boundaries that could potentially create inaccurate matching of SEIFA and CDCB data for some cases.

## Conclusions

This study has mapped the areas of greatest HCV treatment need in SA. Most people diagnosed with HCV were from marginalised sub-populations and clustered in the least economically-resourced areas. Subsequently, it is imperative that initiatives aiming to improve DAAs treatment uptake target socioeconomically disadvantaged and marginalised sub-populations. Indigenous Australians, non-employed people, people who have injected drugs, and people with a history of imprisonment were at greatest risk of HCV infection. The number of non-employed people, young people, and males statistically less likely to be diagnosed with HCV by general practitioners was concerning, with general practitioners pivotal to providing HCV treatment for many people living with HCV in Australia. Although further research is warranted, these findings set forth an imperative for further action aimed at improving DAAs treatment uptake to reduce the burden of HCV for marginalised people, and progress the aim of eliminating HCV as a public health threat.

## Abbreviations

ABS: Australian Bureau of Statistics
CBD: Central Business District
CDCB: The South Australia Government Health Departments Communicable Disease Control Branch
DAAs: Direct acting antiviral medications
HCV: Hepatitis C virus
IDU: Injecting drug use
IER: Australian Bureau of Statistics 2011 Census Socio-economic Index for Economic Resources
PWID: People who inject drugs
SEIFA: Australian Bureau of Statistics 2011 Census Socio-economic Index for Areas
SES: Socio-economic Status
WHO: World Health Organisation
